This article has been retracted.

# Effect of Core Stability Training on Correction and Surface Electronic Signals of Paravertebral in Adolescent Idiopathic Scoliosis

**DOI:** 10.1155/2022/1819606

**Published:** 2022-08-31

**Authors:** Huijian Weng, Qin Li

**Affiliations:** ^1^Guilin Medical University, Guilin, 541004 Guangxi, China; ^2^Affiliated Hospital of Guilin Medical University, Guilin, 541001 Guangxi, China

## Abstract

**Objective:**

To observe the effect of 12-week core stability training on Cobb angle and the ratios of AEMG (averaged EMG) and IEMG (integral EMG) of paravertebral electromyography in thoracic and lumbar segments in adolescent idiopathic scoliosis (AIS) patients and offer a practical-based evidence for the rehabilitation treatment for AIS patients.

**Methods:**

31 AIS female middle school students were randomly divided into an exercise group (*n* = 16, 12 weeks of core stability training, 3 times/week) and AIS group (*n* = 15). In addition, 15 female secondary school students without scoliosis were included as the normal group (the AIS group and normal group did not perform any regular physical exercise throughout the trial period and only receive regular evaluation and guidance). Before and after the experiment, the digital diagnostic equipment of Philips was used to examine the Cobb angle and Noraxon was used to measure the surface EMG signals of the back thoracic and lumbar paravertebral muscles.

**Results:**

Compared with that before training, after 12 weeks of core stability training, the Cobb angle in the exercise group significantly decreased, and the ratio of AEMG (convex/concave) and IEMG (convex/concave) of paravertebral muscles in the thoracolumbar segment significantly decreased (*P* < 0.01, respectively); there was no significant difference in the above indicators in the AIS group before and after the experiment (*P* > 0.05, respectively). After 12 weeks of core stability training, compared with the AIS group, the Cobb angle decreased significantly (*P* < 0.01), and the ratio of AEMG (convex/concave) and IEMG (convex/concave) of paravertebral muscles in thoracolumbar segment decreased significantly (*P* < 0.01, *P* < 0.05). Compared with the normal group, the ratio of AEMG and IEMG of paravertebral muscles in thoracolumbar segment significantly increased (*P* < 0.01) in the AIS group (*P* < 0.01, respectively).

**Conclusions:**

The core stability training can significantly reduce the Cobb angle of AIS and correct the bad posture of scoliosis patients, which may be related to the balance of the electromyographic activities (convex concave side) of paravertebral muscles in AIS patients.

## 1. Introduction

Scoliosis is a kind of skeletal muscle disease with spinal deflection or rotation, which often occurs in the period of sudden growth before puberty. The etiology of most scoliosis patients is unclear. It is called idiopathic scoliosis in medicine, and approximately 80% of scoliosis patients are adolescent idiopathic scoliosis (AIS) [1]. Worldwide, the prevalence of AIS ranges from 0.93% to 12%, and the incidence and severity of spinal curvature in girls are higher than those in boys [2]. With the development of the body, the degree of spinal deformity in AIS patients is increasing, which makes the patients show abnormal posture, such as stooping, hunchback, and high and low shoulders. These images reflect that AIs may have certain effects on clavicular angle, pelvic inclination angle, Cobb angle, and ankle movement angle and even affect the patient's lung function [3]. At present, the pathogenesis of AIS mainly focuses on genetic, biochemical, mechanical, neural, muscular, and physical factors [4]. Recently, some scholars believe that AIS patients have muscle imbalance on both sides of the spine, which can aggravate the development of scoliosis. In addition, the study of Mahaudens and Mousny [5] showed that the activity of convex paravertebral muscle decreased significantly after spinal fusion, but the effect on concave paravertebral muscle was not obvious. And Liu et al. [6] found that electroacupuncture can improve the spine morphology of IS patients by adjusting the paravertebral muscle electromyographic activity. Based on the above literature, the imbalance of paravertebral muscle activity on both sides of the spine may play an important role in the progression of AIS scoliosis.

At present, the treatment methods for IS are usually divided into two types. According to the degree of Cobb angle, surgery is recommended for patients with a Cobb angle > 40°, and conservative treatment is adopted for AIS patients with a Cobb angle less than 40°, which includes wearing auxiliary devices (brace treatment), spinal adjustment treatment, and exercise treatment [7]. However, ensuring the quality of daily life of AIS patients and choosing a more appropriate treatment method have become a problem for more doctors. The rise of exercise therapy also provides a new idea for the conservative treatment of AIS. It is considered to be an important method to maintain spinal function and can effectively prevent the development of scoliosis. For mild patients with a Cobb angle less than 25°, exercise rehabilitation intervention should be carried out as soon as possible [8]. Recent studies have found that compared with traditional training, core stability training is more effective in reducing rotation deformity and pain in AIS patients, suggesting that core stability training is an effective method for early treatment of AIS [9]. In addition, it is reported that 12-week core stabilization exercise significantly reduces the Cobb angle and improves lumbar muscle strength in AIS patients [10]. Therefore, it can be considered that core stability training may have a more positive impact on spine morphology and back muscle strength balance in AIS patients. Based on the above assumptions, the current study compared the changes of the Cobb angle and EMG (electromyography) signals (the ratios of AEMG and IEMG) of thoracic and lumbar paravertebral muscles in AIS patients after 12 weeks of core stabilization exercise and explored the impact of core stability training on back EMG signals (convex/concave) of AIS patients, so as to provide a theoretical basis for core stabilization exercise intervention in AIS patients.

## 2. Object and Method

### 2.1. Research Object

Thirty-one AIS female middle school students with thoracolumbar double curvature were selected and were randomly divided into an exercise group (*n* = 16) and AIS group (*n* = 15, only receiving regular evaluation and guidance); another 15 female middle school students without scoliosis were selected as the normal group. Inclusion criteria were as follows: (1) meet the diagnostic criteria for scoliosis of the international society of spine surgery; (2) Cobb angle (10°-20°); (3) have not received surgical treatment and have no plans for brace treatment in the near future; (4) no motor organ disease; (5) informed consent to this study, voluntary participation, and signing of informed consent. Exclusion criteria were as follows: (1) nonidiopathic scoliosis; (2) there are growth and development disorder; history of nerve, muscle, and bone infection; spirit; etc; (3) obvious deformity of the lower limbs and feet; and (4) had a history of major surgery. All participants signed the informed consent before the trial (in addition, 2 participants stopped the rehabilitation plan for personal reasons and 14 AIS patients in the EG group). There was no significant difference among the three groups before the exercise intervention in terms of age, height, and weight by one-way ANOVA (*P* > 0.05).  Table 1 shows the basic information of the subjects.

### 2.2. Research Methods

#### 2.2.1. Core Stability Training Program

The core stability training program [11] is designed on the basis of previous studies; all participants performed the core stability training for 12 weeks (3 sessions per week, 60 min each session). Each session includes 10 minutes of warm-up and 5 minutes of relaxation (both stretching and posture exercises of large muscle groups) and 45 minutes of core stability exercise intervention. All movements are carried out under the supervision of professional teachers to ensure that all movements are accurate.

Core stability exercises include unstable equipment exercises (such as balance pad and Swiss ball), back bridge exercise, side bridge exercise, prone two-point support, supine bending and supine leg lifting, trunk curling, and cat camel stretching exercises; each type of exercise was conducted in 3 sets of 12 repetitions. During exercise, the polar table monitors the exercise intensity at any time.

#### 2.2.2. Cobb Angle Measurement

The digital diagnostic equipment of Philips was used to examine the whole spine X-ray plain film (posterior anterior position and lateral position) of 44 subjects before and after exercise intervention. For the posterior-anterior position, the patient stands naturally, feet shoulder-width apart, eyes looks straight ahead, and hands are naturally hanging at the sides of the body; for the lateral position, the patient stands naturally, hip and knee joints are fully extended, elbows are fully flexed, hands are making a fist on the clavicle on the same side and avoid it when shooting limbs overlap with the spine.

Cobb angle was measured using Cobb method. The end vertebrae that were the most tilted toward the concave side of the curvature to be measured were determined at the upper and lower ends of the curvature. One line was drawn above the upper end of the vertebra, and the other line was drawn below the lower end of the vertebra. A line was drawn perpendicular to each line, and the angle in which the lines meet was obtained. The Cobb angle was measured by a specialist in rehabilitation medicine.

#### 2.2.3. Paravertebral Electromyography Measurement

Telemetry myoelectric instrument (Noraxon 16) was used to monitor the surface myoelectric activity of paravertebral muscles of patients. The room temperature was required to be 26°C. No strenuous exercise was performed for 24 hours, and no drugs were used one week before the measurement. The patients were familiar with the measurement process and could complete the specified actions as required. The procedure is as follows: the patients take the prone position and paste the electrode and place arms at the sides of the torso in a relaxed state before the experiment. In patients with thoracolumbar double bending AIS, electrode pairs 1 and 3 shall be pasted at 2 cm from the left and right side of the midline of the spine to the corresponding top vertebral plane of the maximum Cobb angle, and electrode pairs 2 and 4 shall be pasted at 2 cm from the left and right side of the midline of the spine to the corresponding top vertebral plane of the minimum Cobb angle; the reference electrodes are placed 6.5 cm away from the parallel outer side of the corresponding test electrode pair. Each patient recorded 4-lead sEMG signals at the same time.

In this study, BST (Biering Sorensen test) was used to measure the paravertebral muscle function of subjects. The BST is the earliest and widely used research method to evaluate the paravertebral muscle function of the lumbar back. The specific operations are as follows: the patient's upper body is exposed in a prone position, and the lower limbs are fixed on the treatment bed with bandages after sticking the electrode sheet. The patient places his arms on the side of the body and his upper body outside the treatment bed. The patient actively exerts force and backs up to the maximum until the patient is tired after hearing the command. Then, the test is stopped and the surface EMG() signal is recorded. Input the surface EMG signal obtained from the test into software (MR3.10) for signal processing, extract the surface EMG index RMS of paravertebral muscle, calculate the ratios of IEMG and AEMG (convex/concave side), and finally carry out statistical analysis.

### 2.3. Statistical Analysis

All experimental data were presented as mean ± standard deviation. SPSS 21.0 statistical software was used for statistical analysis. Paired sample *t*-test was used for the data of the normal group, AIS group, and exercise group before and after the experiment. One-way ANOVA was used for the difference between the groups before and after exercise. The significance level (*α*) was set to *P* < 0.05.

## 3. Results

### 3.1. Effect of Core Stability Training on Paravertebral Electromyography in Patients with AIS

#### 3.1.1. Effect of Core Stability Training on Thoracic Paravertebral Electromyography in Patients with AIS

Table 2 shows that after 12 weeks of core stability training, compared with that before the intervention, the ratio of AEMG (convex/concave) in the thoracic segment in the exercise group significantly decreased by 13.25% (*P* < 0.01), and the ratio of IEMG (convex/concave) significantly decreased by 11.94% (*P* < 0.01). Compared with that before the intervention, the imbalance of concave convex side increased to some extent, but there was no significant difference in the AIS group (the ratio of AEMG: *P* > 0.05; the ratio of IEMG: *P* > 0.05) and there was no statistical difference between the left and right EMG signals in the normal group before and after the experiment (the ratio of AEMG: *P* > 0.05; the ratio of IEMG: *P* > 0.05).

One-way ANOVA showed that before the intervention, there were significant differences among the three groups (AEMG ratio: *F* = 176.978, *P* = 0.000; IEMG ratio: *f* = 100.342, *P* = 0.000). Compared with the normal group, the ratios of AEMG and IEMG were significant higher in the AIS group and exercise group (*P* = 0.000, *P* = 0.000); compared with the AIS group, there was no significant difference in the ratios of AEMG and IEMG in the exercise (*P* = 0.895, *P* = 0.930). After 12 weeks of exercise intervention, there were still significant differences among the three groups (the ratio of AEMG: *F* = 147.547, *P* = 0.000; the ratio of IEMG is as follows: *F* = 86.020, *P* = 0.000). Compared with the normal group, the ratios of AEMG and IEMG were significantly higher (*P* = 0.000, respectively) in the AIS group and exercise group, but compared with the AIS group, the ratios of AEMG and IEMG were significantly lower (*P* = 0.000, respectively) in the exercise group.

#### 3.1.2. Effect of Core Stability Training on Lumbar Paravertebral Electromyography in Patients with AIS

Table 3 shows that after 12 weeks of core stability training, compared with that before the intervention, the ratio of AEMG (convex/concave) of the lumbar segment in the exercise group decreased significantly by 7.97% (*P* < 0.01), and the ratio of IEMG (convex/concave) decreased significantly by 12.12% (*P* < 0.01). In the AIS group, the imbalance of concave convex side increased to some extent, but there was no significant difference (the ratio of AEMG: *P* > 0.05; the ratio of IEMG: *P* > 0.05). Compared with the normal group before the experiment, there was no significant difference between the left and right muscle electrical signals (the ratio of AEMG: *P* > 0.05; the ratio of IEMG: *P* > 0.05).

One-way ANOVA showed that before the exercise intervention, there were significant differences among the three groups (the ratio of AEMG: *F* = 56.436, *P* = 0.000; the ratio of IEMG ratio: *F* = 45.687, *P* = 0.000). Compared with the normal group, the ratios of AEMG and IEMG (convex/concave) in the AIS group and exercise group increased significantly (*P* = 0.000, respectively). Compared with AIS group, there was no significant difference in the ratios of AEMG and IEMG between the exercise group and AIS group (*P* = 0.554, *P* = 0.108). After 12 weeks of core stability training, there were significant differences among the three groups (AEMG ratio: *F* = 43.479, *P* = 0.000; IEMG ratio: *F* = 48.612, *P* = 0.000). Compared with the normal group, the ratios of AEMG and IEMG (convex/concave) in the AIS group and exercise group significantly increased (*P* = 0.000, respectively). Compared with the AIS group, the ratios of AEMG and IEMG (convex/concave) in the exercise group significantly decreased (*P* = 0.024, *P* = 0.003).

### 3.2. Effect of Core Stability Training on Cobb Angle in AIS Patients

Table 4 shows that after 12 weeks of core stability training, compared with that before exercise, the Cobb angle in the exercise group decreased significantly by 27.97% (*P* < 0.01); but there was no significant difference in the AIS group compared with that before the experiment (*P* > 0.05). There was no significant difference in the Cobb angle between the two groups before exercise (*P* > 0.05). After 12 weeks of core stability training, the Cobb angle in the exercise group decreased significantly compared with that in the AIS group (*t* = 3.700, *P* = 0.001).

## 4. Discussion

### 4.1. Effect of Core Stability Training on Cobb Angle in AIS Patients

Core muscle strength training refers to the training of the muscle strength and control ability at the core of the human body, and the core generally refers to the areas below the shoulder and above the hip, including the spine and pelvis. As early in the 1990s, scholars from the United States and other western countries surveyed the trunk muscles; they conducted in-depth research on the trunk muscles from different angles such as sports anatomy and sports biomechanics, put forward the concept of “core muscle group,” and recognized the important role of core muscle strength in maintaining spinal stability and normal posture [12]. Whether a person is in motion or at rest, core muscle strength is considered as a muscle band to enhance the stability of the spine [13]; some scholars also mentioned the definition of core strength, which means that the body attached to the spine, pelvis, hip, and other bones can maintain basic posture, posture stability, and balance regardless of whether the body is at rest or in the motion [14].

The double curvature type AIS patients are selected in this study and the average Cobb angle is15.27 ± 2.66degrees, which belong to mild AIS patients. The AIS patients are subject to 12 weeks of core stability training; during the core muscle strength training, the patients are always in a normal position, and the muscle strength training of the trunk is balanced as far as possible. Therefore, the spine can be ensured to be on the correct force line and can also make the spine in a more stable state through effective core muscle strength training. Research suggests that the transverse abdominal muscle and internal oblique abdominal muscle can not only enhance the stability of the spine and pelvis but also increase the abdominal pressure [13], which can not only change the scoliosis state but also peel off the adhesion of the ligament soft tissue, improve the muscle blood supply, and enhance its elasticity, and the soft tissue and ligament can also be softened. The results of this study showed that after 12 weeks of core stability training, the Cobb angle of AIS patients in the exercise group decreased significantly, and the results are consistent with that of previous scholars [11]. In addition, this study also found that during the 12 weeks of experiment, the Cobb angle of the AIS group increased from 15.71 ± 2.70 degrees to 16.07 ± 2.95, suggesting that AIS patients were at risk of aggravating spinal deformity without any treatment. However, the duration of exercise intervention is very important. Some scholars suggest that exercise therapy for AIS patients should last for at least 6 months or longer, which will have a greater impact on the Cobb angle [15]. Therefore, the follow-up study should extend the intervention time of core stability training and verify the duration of the rehabilitation effect of core stability training on AIS patients.

### 4.2. Effect of Core Stability Training on sEMG Signal of Paravertebral Muscle in Patients with AIS

SEMG is called a biometric technology to test the neuromuscular response during various activities. SEMG signals represent the characteristics of muscle function, provide information about muscle activities, and can be used as an important reference for formulating treatment plans for muscle function diseases [16]. Biopsy study showed that paravertebral muscle structure, protein synthesis, and muscle fiber type composition were abnormal in AIS patients [17]. In the study of the cause and mechanism of scoliosis, the theory of paravertebral muscle abnormality is controversial. However, in the etiological study of AIS, the abnormal distribution of paravertebral muscle electromyography has been confirmed by most scholars that the back muscle activity between the concave and convex sides of the spine is obviously asymmetric. The increase of convex side electromyogram activity and the decrease of concave side electromyogram activity are one of the risk factors for the aggravation of spinal curvature [18]. SEMG can be used as one of the objective examinations to evaluate the back electromyographic activity of scoliosis [19]. Xu et al. [20] found that the proportion distribution of muscle fiber types in paravertebral muscles of AIS patients was unbalanced through the analysis of electromyographic signals of paravertebral muscles on the concave convex side in the back of adolescent scoliosis patients. The larger the Cobb angle, the greater the difference of back muscle strength on the concave convex side, and the more obvious the imbalance. At the same time, Zheng et al. [21] found that there was no significant difference in the EMG activity of the convex/concave side between the younger age group (7-10-year-old group) and the control group, while there were more differences between the older age group (11-14-year-old group) and the control group, which mainly manifested in the convex side. Therefore, they believed that the EMG changes of the paravertebral side were the main results of scoliosis. And the older the age, the longer the course of disease, the greater the Cobb angle, and the greater the load of the convex side muscle to maintain body balance, so the difference of EMG activity is more obvious. Cheung et al. [22] found that the EMG ratio of convex/concave side of scoliosis patients in sitting and standing posture significantly increased, which suggested that the EMG activity of paravertebral muscles might have important reference value for predicting scoliosis. The current study found that the ratios of AEMG and IEMG in the left and right of the back thoracic and lumbar segments in the normal group of female middle school students were close to 1, which showed that the muscle strength of both sides was basically symmetrical. While the ratios of AEMG and IEMG(convex/concave) in the thoracolumbar of 29 AIS patients significantly increased (greater than 1) which indicated that the muscle strength of paravertebral muscles on the concave convex side in the back thoracolumbar segment of AIS female middle school students was unbalanced, which was consistent with the research results of the above scholars.

Previous studies have confirmed that scoliosis interventions can improve the spinal morphology of scoliosis patients by balancing paravertebral muscle electromyography. Liu et al. [6] found that after the electroacupuncture plus chiropractic intervention, the motor potential amplitude of scoliosis patients increased in concave side and decreased in convex side (before the intervention, the concave side decreased and the convex side increased), and the Cobb angle significantly improved, which suggested that electroacupuncture chiropractic treatment has a significant adjustment effect on scoliosis patients. In addition, Ko et al. [23] found that asymmetric spinal stability exercises can significantly increase the average RMS and peak amplitude of the concave side in the paravertebral muscle, and the Cobb angle of the patients significantly decreased. They believed that asymmetric spinal stability exercises can improve the severity of scoliosis by strengthening the concave paravertebral muscle. BST is the earliest and widely used research method to evaluate the function of lumbar paravertebral muscle [20]. Through the BST experiment, the current study found that after 12 weeks of core stability training, the ratios of IEMG and AEMG (convex/concave) in paravertebral muscles of thoracic and lumbar segments in the exercise group significantly decreased, but the ratio was still higher than 1, and there was still significant difference compared with the normal control group, which indicated that 12 weeks of core stability training can effectively balance the EMG activity in the convex concave side of AIS patients, but it cannot be completely improved; future research needs to extend the intervention time of core stability training to verify its effect. It is believed that the imbalance of paravertebral muscle electromyographic activity is one of the risk factors for the aggravation of spinal curvature [24]. Therefore, the core stability training to balance the EMG activity(convex/concave) of paravertebral muscles may be beneficial to the improvement of spinal deformity in patients with scoliosis in this study may be related to the decrease of Cobb angle in AIS patients, and the specific mechanism needs to be further studied.

## 5. Summary

12-week core stabilization training can effectively improve the spinal deformity of AIS patients and balance the EMG activity of the convex and concave sides of patients which may be related to the release of the back muscles and the activation of the weak side muscles by core stabilization training in patients with AIS, but it cannot be completely improved. In order to verify its effect, later studies need to extend the core stabilization training intervention time.

## Figures and Tables

**Table 1:** Physical characteristics of subjects (*x* ± *s*).

	*n*	Age (year)	Height (m)	Weight (kg)
Normal group	15	13.34 ± 1.08	1.56 ± 0.02	47.76 ± 2.13
AIS group	14	13.87 ± 0.96	1.57 ± 0.01	48.02 ± 1.25
Exercise group	15	13.15 ± 0.47	1.56 ± 0.03	48.32 ± 1.98

**Table 2:** Changes of sEMG signal in thoracic paravertebral muscle of AIS patients in BST (*x* ± *S*, *μV*/*s*).

sEMG	Group	Before	After	*t*	*P*
The ratio of AEMG (convex/concave)	Exercise group	1.51 ± 0.08^∗∗^	1.32 ± 0.10^##^^∗∗^^∆∆^	7.893	0.000
	AIS group	1.48 ± 0.11^∗∗^	1.50 ± 0.08^∗∗^	-0.575	0.576
	Normal group	1.02 ± 0.04	1.01 ± 0.03	0.503	0.623

The ratio of IEMG (convex/concave)	Exercise group	1.39 ± 0.08^∗∗^	1.19 ± 0.11^##^^∗∗^^∆∆^	11.037	0.000
	AIS group	1.37 ± 0.12^∗∗^	1.38 ± 0.09^∗∗^	-0.595	0.562
	Normal group	1.00 ± 0.04	1.01 ± 0.05	-0.321	0.576

Note: ^##^*P* < 0.01 comparison before and after experiment; ^∗∗^*P* < 0.01 vs. normal group; ^∆∆^*P* < 0.01, vs. the AIS group.

**Table 3:** Changes of sEMG signal in the lumbar paravertebral muscle of AIS patients in BST (*x* ± *S*, *μV*/*s*).

sEMG	Group	Before	After	*t*	*P*
The ratio of AEMG (convex/concave)	Exercise group	1.38 ± 0.10^∗∗^	1.27 ± 0.13^##^^∗∗^^∆^	4.119	0.001
	AIS group	1.33 ± 0.14^∗∗^	1.37 ± 0.12^∗∗^	-1.836	0.089
	Normal group	1.01 ± 0.05	1.00 ± 0.03	1.424	0.176

The ratio of IEMG (convex/concave)	Exercise group	1.32 ± 0.12^∗∗^	1.16 ± 0.10^##^^∗∗^^∆∆^	5.520	0.000
	AIS group	1.26 ± 0.12^∗∗^	1.29 ± 0.08^∗∗^	-0.880	0.395
	Normal group	1.00 ± 0.03	1.01 ± 0.04	-0.269	0.792

Note: ^##^*P* < 0.01, comparison before and after experiment; ∗∗*P* < 0.01, vs. the normal group; ^∆∆^*P* < 0.01 vs. the AIS group.

**Table 4:** Results of Cobb angle pre and post the core stabilization training in AIS (*x* ± *s*).

Group	*n*	Before	After	*t* value	*P* value
AIS group	14	15.71 ± 2.70	16.07 ± 2.95	-1.161	0.266
Exercise group	15	14.87 ± 2.64	12.40 ± 2.47^##*ΔΔ*^	6.788	0.000

Note: ^##^*P* < 0.01, comparison before and after experiment; *^ΔΔ^P* < 0.01, vs. the control group.

## Data Availability

The raw data supporting the conclusions of this article will be made available by the authors, without undue reservation.
